RETRACTED

# Meta-Analysis of the Relationship between the Prognosis of Acute Cerebral Infarction Intravenous Lysis and Cerebral Microbleeds Based on Intelligent Medical Care

**DOI:** 10.1155/2022/4329318

**Published:** 2022-08-29

**Authors:** Kui Duan, Yufang Wu

**Affiliations:** ^1^Neurology Department Cerebrovascular Disease, People's Hospital of Dejiang, Tongren, Guizhou 565200, China; ^2^Neurology, Daqing People's Hospital, Daqing, Heilongjiang, China

## Abstract

The accelerated pace of life leads to people's unhealthy living habits such as irregular diet, irregular work and rest, and fatigued work. The incidence of acute cerebral infarction (ACI) is increasing year by year. Intravenous thrombolysis is the best solution for clinical treatment of ACI, but intravenous thrombolysis increases the risk of cerebral microbleeds and even seriously damages the brain of patients. It is crucial to analyze the relationship between intravenous thrombolysis of ACI and cerebral microbleeds. Using intelligent medical methods such as BP neural network (BPNN), meta-analysis was carried out on the prognosis of ACI intravenous thrombolysis and cerebral microbleeds, and the basic data indicators, living habits indicators, and ACI intravenous thrombolysis indicators of ACI patients were analyzed. The experimental results showed that the odds ratios (OR) of systolic blood pressure before ACI intravenous thrombolysis, blood glucose concentration after ACI intravenous thrombolysis, diastolic blood pressure before ACI intravenous thrombolysis, and diastolic blood pressure after ACI intravenous thrombolysis on cerebral microbleeds after ACI intravenous thrombolysis were 0.97, 0.44, 0.13, and 0.07, respectively. Long-term intravenous thrombolysis with ACI, high systolic blood pressure after NIHSS thrombolysis with high scores, and blood glucose concentration before thrombolysis had OR >1, which were risk factors for cerebral microbleeds after intravenous thrombolysis with ACI. Therefore, paying attention to the risk factors of cerebral microbleeds during ACI intravenous thrombolysis can effectively reduce cerebral microbleeds after ACI intravenous thrombolysis and improve the treatment efficiency of ACI patients.

## 1. Introduction

With the change of people's lifestyle, ACI has become one of the most common clinical diseases. ACI is caused by partial brain tissue necrosis or ischemia. ACI treatment is difficult to treat, and the prognosis of treatment is variable. It is by far the second leading cause of death, with 6% of global deaths from ACI. Since 1996, alteplase has been used in the clinical diagnosis and treatment of ACI by intravenous thrombolysis, and good therapeutic effects have been achieved, but there have also been many prognostic problems of intravenous thrombolysis of ACI, of which cerebral microbleeds are the most common problem. If the cerebral hemorrhage is not treated in time, the patient will die of cerebral hemorrhage. With the development of intelligent medical care, the use of BPNN and classification algorithm can realize the predictive analysis of medical factors, and the relationship between ACI intravenous thrombolysis and cerebral microbleeds can be effectively analyzed in conjunction with meta-analysis. To find out the risk factors of cerebral microbleeds after intravenous thrombolysis of ACI, effectively reduce the secondary symptoms of cerebral microbleeds after intravenous thrombolysis of ACI, and improve the degree of treatment of ACI, this paper has research significance.

RETRACTED

ACI intravenous thrombolysis will cause certain damage to the brain of patients. Some researchers have analyzed the relationship between ACI intravenous thrombolysis and cerebral microbleeds. Among them, Liang Y.'s study mainly analyzed the relationship between ACI intravenous thrombolysis and the bleeding volume of cerebral microbleeds, so as to achieve the purpose of reducing cerebral hemorrhage [1]. Alaa et al. have studied some risk factors for cerebral microbleeds after ACI intravenous thrombolysis, including age and blood pressure [2]. Zhai et al. divided the patients with cerebral microbleeds after ACI intravenous thrombolysis into two groups and analyzed the factors causing cerebral microbleeds through the comparison between groups and logistic regression [3]. Pan et al. conducted a correlation analysis of cerebral microbleeds in patients with special diagnosis such as gender, age, and medical history records [4]. Dong et al.'s study pointed out that different races are related to cerebral microbleeds after ACI intravenous thrombolysis [5]. Through the factor analysis of ACI intravenous thrombolysis and cerebral microbleeds, some indicators that cause cerebral microbleeds can be found, but there is a lack of intelligent analysis methods.

The meta-analysis based on intelligent medicine can effectively analyze the relevant factors of medical problems, and the relationship between ACI intravenous thrombolysis and cerebral microbleeds is studied through the meta-analysis of intelligent medicine. Among them, Papadopoulos A. used meta-analysis of ACI intravenous thrombolysis and cerebral microbleeds and judged the influencing factors by comparative odds ratio [6]. Tomohiro et al. used intelligent medical technology to analyze the related factors of the prognosis of ACI intravenous thrombolysis and determined the influencing factors through the meta-analysis of related factors and cerebral microbleeds [7]. Xia et al.'s experiment applied the meta-analysis of intelligent medicine to the study of ACI intravenous thrombolysis and cerebral microbleeds and concluded that the influencing indicators are hypertension and elevated systolic blood pressure before ACI intravenous thrombolysis [8]. In Meng et al.'s study, a meta-analysis was conducted on clinical diagnosis and treatment factors and cerebral microbleeds of ACI intravenous thrombolysis, and the related factors were obtained [9]. Zhou et al. could reduce the factors of cerebral microbleeds after ACI intravenous thrombolysis through Bayesian meta-analysis [10]. Meta-analysis based on intelligent medical can well study the relationship between ACI intravenous thrombolysis and cerebral microbleeds, but the intelligent medical technology used is not optimal.

RETRACTED

In this paper, the meta-analysis method of intelligent medicine is used to study the prognosis of ACI intravenous thrombolysis and the risk factors of cerebral microbleeds. The innovations of this paper are as follows: (1) A research on the combination of intelligent medicine and meta-analysis is carried out. (2) The ACI patients were divided into a case group and a control group according to whether the symptoms of cerebral microbleeds occurred after receiving intravenous thrombolysis, and the related factors were analyzed for the two groups.

## 2. Meta-Analysis Method of the Relationship between the Prognosis of ACI and Intravenous Lysis and Cerebral Microbleeds Based on Intelligent Medicine

In this paper, a meta-analysis of intelligent medical treatment was carried out on the prognosis of ACI intravenous thrombolysis and cerebral microbleeding, and the factors of cerebral microbleeding after ACI intravenous thrombolysis were predicted and analyzed by neural network and other technologies, and the risk factors related to cerebral microbleeding were calculated by meta-analysis [11]. The meta-analysis model of the prognosis of ACI intravenous lysis and cerebral microbleeds is shown in Figure 1.

It can be seen from Figure 1 that ACI intravenous thrombolysis may cause cerebral microbleeds, and the methods to analyze the risk factors for cerebral microbleeds are intelligent medicine and meta-analysis. The methods of meta-analysis include Peto method, Mantel-Haenszel method, and migration analysis.

### 2.1. BPNN

#### 2.1.1. Neurons

BPNN is a kind of artificial neural network; artificial neural network is the process of simulating biological neural computing; axons and dendrites in biological nerves are abstracted as neuron nodes of BPNN. It can be a good analysis of the prognosis of acute cerebral infarction and the related factors of cerebral microbleeds [12]. In the BPNN, the neuron is the most basic processing unit and the most basic computing unit. The calculation process of the BPNN is realized by the information transmission between the neurons. The neuron model is shown in Figure 2.

RETRACTED

In Figure 2, the BP neuron needs to process many input signals. Let the input signal of the neuron be (*x*_1_, *x*_2_, ⋯, *x*_*n*_), and let the connection weight between the neuron and the input signal be *V*=(*v*_1_, *v*_2_, ⋯, *v*_*n*_), where *θ* represents the threshold of the neuron. The signal processing process is the sum of the product of the input signal and the connection weight, and the threshold *θ* of the neuron is subtracted after processing [13]. The result after neuron processing is

(1) $$\begin{array}{c} s=\sum_{k=1}^{n}v_{k}x_{k}. \end{array}$$

In formula (1), *x*_*k*_ represents the *k*th input signal.

Then the result of neuron processing is passed into function *g* and finally output; function *g* is the sigmoid function:

(2) $$\begin{array}{c} g\left(s\right)=\frac{1}{1+e^{-s}}. \end{array}$$

#### 2.1.2. BPNN Model

Due to the characteristics of information transmission, BPNN has excellent computing ability and dynamic learning ability [14]. BPNN has unique information transmission ability. Its core information transmission process is the back-propagation of errors. Through layer-by-layer feedback, neurons are continuously adjusted to change the structure of the neural network, so that the BPNN's actual output is close to the expected output. BPNN is a classic three-layer network structure, and its structure is shown in Figure 3.

As can be seen from Figure 3, the BPNN has two modes of information dissemination, positive and negative. The propagation process is divided into forward propagation of information and back-propagation of errors.

#### 2.1.3. BPNN Learning Process

The learning process of the BPNN is error reduction process. When the BPNN performs the feedback adjustment of the error, it changes the structure of the BP neural network by changing the neuron weights, thereby changing the output, and finally, the error between the actual output of the BPNN is within an acceptable range [15].

Therefore, the error feedback of the BPNN is the key to the learning of the BPNN. The error formula of the BPNN is expressed as

(3) $$\begin{array}{c} E=\frac{1}{2}\sum_{k}{\left(g_{k}^{a}-g_{k}^{b}\right)}^{2}. \end{array}$$

If the connection weight is (*v*_11_, *v*_12_, ⋯, *v*_*ij*_, ⋯), then the BPNN error can be represented by a weight vector. The learning process of the BPNN is the process of making the error smaller. Until the error reaches an acceptable range, the learning process of the BP network is essentially a problem of finding the minimum solution [16].

RETRACTED

The error feedback mechanism of the BPNN is to use the gradient descent method to solve the minimum value of the error. The solving process is as follows:

(4) $$\begin{array}{c} \nabla E=\nabla g\left(v_{11},v_{12},\cdots v_{ij}\right)={\left[\frac{\partial g}{\partial v_{11}},\frac{\partial g}{\partial v_{12}},\cdots ,\frac{\partial g}{\partial v_{ij}}\right]}^{T}. \end{array}$$

In formula (4), *T* represents transposition.

It can be seen from formula (4) that finding the minimum value of the error is essentially the same process as finding the minimum value of *∂g*/*∂v*_*ij*_. Let the input layer, the hidden layer, and the output layer be represented by *P*, *Q*, and *R*, respectively. The numbers of elements are *p*, *q*, and *r*, respectively.

The partial derivative of the output layer error function is expressed as

(5) $$\begin{array}{c} \frac{\partial E}{\partial v_{jk}}=\frac{\partial E}{\partial g_{j}}\cdot \frac{\partial g_{j}}{\partial v_{jk}}. \end{array}$$

The expression of the error has been declared in formula (3), and formula (3) and formula (5) are sorted out:

(6) $$\begin{array}{c} \frac{\partial E}{\partial g_{k}}=-{\left(g_{k}^{a}-g_{k}^{b}\right)}^{2}. \end{array}$$

The output of the hidden layer neurons is expressed as

(7) $$\begin{array}{c} g_{j}=\text{sig}\left(\sum_{i}v_{ij}Q_{j}\right). \end{array}$$

In formula (7), *i* represents the *i*th input layer neuron. *Q*_j_ represents the *j*th hidden layer neuron.

The hidden layer partial derivative is expressed as

(8) $$\begin{array}{c} \frac{\partial g_{j}}{\partial v_{ij}}=\text{sig}{}^{\prime }\left(\sum_{i}v_{ij}Q_{j}\right)Q_{j}. \end{array}$$

Integrating equation (5), equation (6), and equation (8), we get

(9) $$\begin{array}{c} \frac{\partial E}{\partial v_{jk}}=\phi_{k}^{r}Q_{j}. \end{array}$$

In (9), *ϕ*_*k*_^*r*^ represents the learning factor of the output layer.

The learning factor *ϕ*_*k*_^*r*^ of the output layer is expressed as

(10) $$\begin{array}{c} \phi_{k}^{r}=-\left(g_{k}^{a}-g_{k}^{b}\right)\text{sig}{}^{\prime }\left(\sum_{j}v_{jk}Q_{j}\right). \end{array}$$

In formula (10), sig represents a regression analysis function.

As with the learning factor of the output layer, the learning factor of the hidden layer can be calculated as

(11) $$\begin{array}{c} \phi_{j}^{q}=-\left(g_{j}^{a}-g_{j}^{b}\right)\text{sig}{}^{\prime }\left(\sum_{i}v_{ij}Q_{i}\right). \end{array}$$

### 2.2. Meta-Analysis

Meta-analysis is a statistical analysis method. It mainly collects and sorts out the relevant factors to find out the relationship between the relevant factors and the research questions. It can well analyze the relationship between the prognosis of acute cerebral infarction and the cerebral microbleeds.

RETRACTED

Meta-analysis can be divided into random-effects model and fixed-effects model according to different statistical classifications [17]. The fixed-effects model sets the hypothetical true value of the research experiment to be the same, while the random-effects model assumes that the true value of the experiment is different. The random-effects model is the most widely used model in meta-analysis, and the meta-analysis structure is shown in Figure 4.

Common calculation methods for meta-analysis include Peto method and Mantel-Haenszel method.

#### 2.2.1. Peto Method

In the study of analyzing the prognosis of ACI intravenous lysis and cerebral microbleeds, let *e* be the number of cerebral hemorrhages caused by a particular variable in the experimental group, let *f* be the total number of cerebral hemorrhages caused by a particular variable in the experimental group, and let *g* be the number of cerebral hemorrhages caused by a particular variable in the control group; *h* is the total number of particular variables in the control group [18].

Then the expected formula for the occurrence of each factor in the experimental group is expressed as

(12) $$\begin{array}{c} E_{ei}=\frac{n_{1i}\left(e_{i}+g_{i}\right)}{N_{i}}. \end{array}$$

In formula (12), *N* represents the number of factors.

The variance of each factor is expressed as

(13) $$\begin{array}{c} D_{i}=\frac{n_{1i}n_{2i}\left(e_{i}+g_{i}\right)\left(f_{i}+h_{i}\right)}{N_{i}^{2}\left(N_{i}-1\right)}. \end{array}$$

In formula (13), *D*_i_ represents the variance of the *i*th factor.

The formula for the odds ratio of each factor is

(14) $$\begin{array}{c} {\text{OR}}_{i}=\exp\left(\frac{e_{i}-E_{ei}}{D_{i}}\right). \end{array}$$

The effect values for all factors are

(15) $$\begin{array}{c} \text{OR}=\exp\left(\frac{\sum D_{i}\ln\left({\text{OR}}_{i}\right)}{\sum D_{i}}\right). \end{array}$$

In formula (15), “exp” represents an exponential function with base *e*.

#### 2.2.2. Mantel-Haenszel Method

Calculate the odds ratio for each factor:

(16) $$\begin{array}{c} {\text{OR}}_{j}=\frac{e_{j}g_{j}}{f_{j}h_{j}}. \end{array}$$

To find the standard deviation of the odds ratio of each factor, the formula is as follows:

(17) $$\begin{array}{c} S=\sqrt{\frac{1}{e_{j}}+\frac{1}{f_{j}}+\frac{1}{g_{j}}+\frac{1}{h_{j}}}. \end{array}$$

Find the weight of each factor:

(18) $$\begin{array}{c} w_{j}=\frac{f_{j}g_{j}}{N_{j}}. \end{array}$$

In formula (18), w_*j*_ represents the weight of the *j*th factor.

RETRACTED

The odds ratio of each factor and its corresponding weight are added together to obtain the overall odds ratio.

#### 2.2.3. Offset Analysis

Offset analysis is a comprehensive analysis of the experimental odds ratios and weights of the control group and the experimental group. It is mainly expressed in the form of a funnel diagram, which can visually display the odds and weights of each factor.

The funnel plot mainly analyzes the logarithm of the effect value and the scatter plot of the standard error. Generally, OR or RR is used as the effect value for analysis. The structural model of the funnel plot is shown in Figure 5.

In Figure 5, the analysis principle of the funnel plot is as follows: when the precision of the effect size tends to rise as the number of samples increases, the curve becomes high and narrow, and it finally tends to a point, forming an inverted funnel shape [19]. The larger the sample size and the higher the precision, the higher the factor, so the last point is the result of the study.

When the meta-analysis has statistical significance, the offset calculation is required, and the calculation formula is as follows:

(19) $$\begin{array}{c} N_{e}={\left(\frac{\sum a_{i}}{a_{e}}\right)}^{2}-k. \end{array}$$

### 2.3. Support Vector Machine Technology

Support vector machines are widely used in classification and regression prediction [20]. Among the risk elements for analyzing the relationship between the prognosis of ACI intravenous lysis and cerebral microbleeds, the support vector machine can accurately classify the types of various influencing elements, which provides important help for the subsequent calculation of the correlation of the influencing elements. Support vector machines can handle nonlinear classification problems well, and the support vector machine model is shown in Figure 6.

In Figure 6, the support vector machine has a good classification effect, and the different categories of factors affecting the prognosis of ACI intravenous lysis and cerebral microbleeds are separated according to the characteristic interval. The fundamental idea is to find two categories. The formula for the classification surface is expressed as

(20) $$\begin{array}{c} u^{T}x+v=0. \end{array}$$

In formula (20), (*u*=*u*_1_, *u*_2_, ⋯, *u*_*n*_) is the center line of the classification surface and is also the basis for the classification of two different factors, and *v* represents the straight-line distance from the classification surface to the origin.

The classification surface is determined by two variables *u* and *v*. The formation and scope of the classification surface are determined by *u* and *v*. The classification surface can be expressed as (*u*, *v*). Then the distance between the prognosis of ACI intravenous lysis and the related factors of cerebral microbleeds to the classification surface can be expressed as

(21) $$\begin{array}{c} d=\frac{\left|u^{T}x+v\right|}{\left|u\right|}. \end{array}$$

In formula (21), *d* represents the distance from the correlation factor to the classification surface.

RETRACTED

When dealing with the classification problem of linearly correlated factors, the correlated factors can be represented by (*x*, *y*) ∈ *R*; then the following equation holds:

(22) $$\begin{array}{c} \left\{\begin{array}{c} u^{T}x+v\geq +1,y=+1,\\ u^{T}x+v\leq -1,y=-1. \end{array}\right) \end{array}$$

Then the distance from a correlation factor to the classification surface can be expressed as

(23) $$\begin{array}{c} d=\frac{1}{\left|u\right|}. \end{array}$$

Maximize the separation of the classification surfaces, that is, maximize distance *d* in formula (23):

(24) $$\begin{array}{c} \underset{u,v}{\max}\frac{1}{\left|u\right|}. \end{array}$$

Formula (24) can be transformed into a binary equation solving problem, and the expression after transformation is

(25) $$\begin{array}{c} \underset{u,v}{\min}\frac{1}{2}{\left|u\right|}^{2}. \end{array}$$

## 3. Meta-Analysis Experiment on the Relationship between the Prognosis of ACI Intravenous Lysis and Cerebral Microbleeds Based on Intelligent Medicine

### 3.1. Experimental Data

At present, the first choice for clinical treatment of acute cerebral infarction is intravenous thrombolysis, but intravenous thrombolysis may cause cerebral microbleeds in patients, The experiment will use meta-analysis of the relationship between the prognosis of ACI and cerebral microbleeds based on intelligent medical treatment. When the experiment is carried out, it is necessary to select the experimental object.

The experimental data comes from 100 ACI patients from 2019 to 2020, 40 girls and 60 boys, all diagnosed by CT and other means. The selection criteria for the experimenters were as follows: age less than 80 years, onset time less than 6 hours, NIHSS score greater than 4, and nonintracerebral hemorrhage confirmed by medical imaging. The exclusion criteria of the experimenter were as follows: history of cerebral hemorrhage, other affecting diseases, and unstable blood sugar and blood pressure.  Table 1 shows the information of the experimenter.

Intravenous thrombolysis was performed on the experimenters, and 0.9 mg of the drug was injected per kg of body weight, and the maximum cannot exceed 90 mg, which was injected intravenously.

Investigate and count the indicators of cerebral microbleeds which affect the prognosis of ACI by intravenous lysis, and make statistics on the patients' living habits, the time of intravenous thrombolysis, and other disease characteristics to influence the prognosis of ACI by intravenous lysis. The data indicators of cerebral microbleeds are shown in Table 2.

RETRACTED

After intravenous thrombolysis in 100 ACI patients, the case group was made up of ACI patients who had cerebral microbleeds, and the ACI patients without cerebral hemorrhage were set as the control group. Through meta-analysis of case group and control group, the relationship between the prognosis of ACI intravenous lysis and cerebral microbleeds was found out.

### 3.2. Meta-Analysis of the Prognosis of ACI by Intravenous Lysis and Cerebral Microbleeds

In order to analyze the relationship between the prognosis of ACI intravenous lysis and cerebral microbleeds, it is necessary to count the characteristics of the control group and the case group. The distribution of cerebral microbleeds in ACI is shown in Figure 7.

From the distribution of the number of microbleeds in Figure 7, it can be seen that, among male patients, 12 patients developed cerebral hemorrhage symptoms after intravenous thrombolysis, and the most common people were 58–62 years old and 66–70 years old. Among the female patients, 8 had symptoms of cerebral hemorrhage. Overall, the rate of cerebral microbleeds in ACI was 20%.

#### 3.2.1. Factors Associated with Cerebral Hemorrhage following ACI Intravenous Thrombolysis

Univariate analysis was performed on the influencing indicators, and the *P* value was used to determine whether the indicators were statistically significant.  Table 3 shows the basic variables of cerebral hemorrhage following ACI intravenous thrombolysis.

The analysis of ACI intravenous thrombolysis factors for cerebral hemorrhage after ACI intravenous thrombolysis is shown in Table 4.

In Tables 3 and 4, the *P* value is the logistic regression analysis. When *P* < 0.05, the single-factor influencing indicators of cerebral hemorrhage after ACI intravenous thrombolysis are ACI thrombolysis time, NIHSS score, systolic blood pressure after thrombolysis, and blood glucose concentration before thrombolysis.

Multivariate analysis was performed on the single-factor influencing indexes of cerebral hemorrhage after ACI intravenous thrombolysis, and the analysis results are shown in Table 5.

The results in Table 5 show that long-term ACI thrombolysis, high NIHSS score, high systolic blood pressure after thrombolysis, and high blood glucose concentration before thrombolysis are risk factors for cerebral hemorrhage after intravenous ACI thrombolysis.

#### 3.2.2. Heterogeneity Analysis of Cerebral Hemorrhage after ACI Intravenous Thrombolysis

The factors were as follows: systolic blood pressure before intravenous thrombolysis of ACI (factor 1), diastolic blood pressure before intravenous thrombolysis of ACI (factor 2), diastolic blood pressure after intravenous thrombolysis of ACI (factor 3), and blood glucose concentration after intravenous thrombolysis of ACI (factor 4). The analysis results of the *Q* test and the *I*^2^ test for the four factors are shown in Figure 8.

RETRACTED

From the analysis in Figure 8, it can be seen that the *Q* tests of the four factors tested are all greater than 0.1, and the *I*^2^ test is less than 25%. There was no clear heterogeneity among the four factors tested as shown. It is necessary to calculate the odds ratio (OR) using the Peto method to determine the relationship of various factors to cerebral microbleeds after ACI intravenous thrombolysis in intelligent medical care.

*(1) Systolic Blood Pressure before ACI Intravenous Thrombolysis and Blood Glucose Concentration after ACI Intravenous Thrombolysis*. Patients were grouped for ACI intravenous thrombolysis based on intelligent medicine and the odds ratio weight of each group were observed and recorded. The systolic blood pressure before ACI intravenous thrombolysis and the blood glucose concentration advantage ratio after ACI intravenous thrombolysis are shown in Figure 9.

In Figure 9(a), the best predominant value is the first group of systolic blood pressure before ACI intravenous thrombolysis, followed by the first group of blood glucose concentration after ACI intravenous thrombolysis. In (b), the highest weight is in the third group of systolic blood pressure before ACI intravenous thrombolysis, followed by the third group of blood glucose concentration after ACI intravenous thrombolysis. The mean odds ratio for systolic blood pressure before intravenous thrombolysis with ACI was 0.97, and the mean odds ratio for blood glucose concentration after intravenous thrombolysis with ACI was 0.44. OR <1; systolic blood pressure before ACI intravenous thrombolysis and blood glucose concentration after ACI intravenous thrombolysis had no significant difference in intracerebral hemorrhage after ACI intravenous thrombolysis.

*(2) Diastolic Blood Pressure before ACI Intravenous Thrombolysis and Diastolic Blood Pressure after ACI Intravenous Thrombolysis*. Seven groups of patients were treated with ACI intravenous thrombolysis based on intelligent medicine. The advantages of diastolic blood pressure before ACI intravenous thrombolysis and diastolic blood pressure after ACI intravenous thrombolysis on cerebral microbleeds are shown in Figure 10.

In Figure 10, the weight of the diastolic blood pressure before ACI intravenous thrombolysis was the highest in the third group, being 50%, and the corresponding dominance value was 0.06. The third group had the highest weight of diastolic blood pressure after ACI intravenous thrombolysis, with a weight of 44%, and the corresponding odds value was 0.08. The mean odds ratio for diastolic blood pressure before intravenous thrombolysis with ACI was 0.13, and the mean odds ratio for diastolic blood pressure after intravenous thrombolysis with ACI was 0.07. OR <1; the diastolic blood pressure before ACI intravenous thrombolysis and the diastolic blood pressure after ACI intravenous thrombolysis had no significant difference in intracerebral hemorrhage after ACI intravenous thrombolysis.

RETRACTED

### 3.3. Experimental Analysis

From the experimental data, we can obtain the odds ratio of cerebral hemorrhage factors after ACI intravenous thrombolysis. The blood glucose concentration after intravenous thrombolysis with ACI, the diastolic blood pressure before intravenous thrombolysis with ACI, and the diastolic blood pressure after intravenous thrombolysis with ACI were recorded as factors 1 to 8, and the advantage ratios of all factors are shown in Figure 11. OR >1 means it is a risk factor for cerebral hemorrhage after ACI intravenous thrombolysis, OR = 1 means there is no relationship between the two, and OR <1 means it is not a risk factor for cerebral hemorrhage after ACI intravenous thrombolysis.

## 4. Discussion

ACI mainly causes cerebral hypoxia death through vascular blockage. The most common and effective treatment is ACI intravenous thrombolysis, but ACI intravenous thrombolysis is often accompanied by cerebral microbleeds. The causes of cerebral microbleeds after intravenous thrombolysis in ACI by means of intelligent medicine are meta-analyzed.

## 5. Conclusions

In this paper, through meta-analysis of the relationship between the prognosis and cerebral microbleeds of ACI intravenous thrombolysis based on intelligent medicine and through univariate analysis, multivariate analysis, and heterogeneity analysis of the influencing factors of statistical investigation, the experimental results show the following: (1) long-term timed ACI intravenous thrombolysis, high systolic blood pressure after NIHSS thrombolysis with high scores, and high blood glucose concentration before thrombolysis are the main factors that cause cerebral microbleeds with ACI intravenous thrombolysis. (2) There was no heterogeneity among systolic blood pressure before ACI intravenous thrombolysis, blood glucose concentration after ACI intravenous thrombolysis, diastolic blood pressure before ACI intravenous thrombolysis, and diastolic blood pressure after ACI intravenous thrombolysis. The OR values for cerebral microbleeds after ACI intravenous thrombolysis were 0.97, 0.44, 0.13, and 0.07, and it is clear that all are less than 1. These four factors were not risk factors for cerebral microbleeds after ACI intravenous thrombolysis. Therefore, prolonged ACI intravenous thrombolysis, high systolic blood pressure after NIHSS thrombolysis with a high score, and high blood glucose concentration before thrombolysis are risk factors for cerebral microbleeds with ACI intravenous thrombolysis. Attention should be paid to these during intravenous ACI thrombolysis. Risk factors can be effective in reducing cerebral microbleeds. However, the factors tested in this paper cannot comprehensively summarize all the factors that cause cerebral microbleeds after ACI intravenous thrombolysis. Therefore, expanding the research on the factors of cerebral microbleeds after ACI intravenous thrombolysis will be the direction of future research.

RETRACTED

## Figures and Tables

**Figure 1:** The meta-analysis model of the prognosis of ACI intravenous lysis and cerebral microbleeds.

**Figure 2:** Neuron model diagram.

**Figure 3:** Structure diagram of BPNN.

**Figure 4:** Meta-analysis structure diagram.

**Figure 5:** Funnel chart.

**Figure 6:** Support vector machine model diagram.

**Figure 7:** The distribution of the number of people with cerebral microbleeds in ACI. (a) Male; (b) female.

**Figure 8:** Heterogeneity analysis of *Q* test and *I*^2^ test.

**Figure 9:** Odds ratio of systolic blood pressure before ACI intravenous thrombolysis and blood glucose concentration after ACI intravenous thrombolysis. (a) Dominance value. (b) Weight.

**Figure 10:** Odds ratio of diastolic blood pressure before ACI intravenous thrombolysis and diastolic blood pressure after ACI intravenous thrombolysis. (a) Dominance value. (b) Weight.

**Figure 11:** Odds ratio plot for all factors.

**Table 1:** Basic data of experimenters.

Basic information	Personnel data
Gender {*n* (%)}	
Male	60 (60.0%)
Female	40 (40.0%)
Age {(*X* ± *S*) years}	60.0 ± 10.0
Weight {(*X* ± *S*) kg}	64.1 ± 9.7
Height {(*X* ± *S*) cm}	168.6 ± 8.8

**Table 2:** Data indicators of cerebral microbleeds affecting the prognosis of ACI by intravenous lysis.

Indicator classification	Impact indicator
Basic data indicators	Age
	Gender

Medical history indicators	Hypertension
	Diabetes

Lifestyle indicators	Smoking
	Drinking

ACI thrombolytic index	ACI thrombolysis time
	NIHSS score
	Systolic blood pressure before ACI thrombolysis
	Systolic blood pressure after ACI thrombolysis
	Diastolic blood pressure before ACI thrombolysis
	Diastolic blood pressure after ACI thrombolysis
	Blood glucose concentration before ACI thrombolysis
	Blood glucose concentration after ACI thrombolysis

RETRACTED

**Table 3:** Analysis of basic factors of cerebral hemorrhage after ACI intravenous thrombolysis.

Group	Age	Male	Female	Hypertension	Diabetes	Smoking	Drinking
Case group (20 people)	60.0 ± 10.0	12	8	8	5	10	6
Control group (80 people)	60.0 ± 10.0	48	32	25	24	30	15
*P* value	0.260	0.512	0.512	0.618	0.582	0.555	0.282

**Table 4:** Analysis of ACI intravenous thrombolysis factors for cerebral hemorrhage after ACI intravenous thrombolysis.

Factor	Case group (20 people)	Control group (80 people)	*P* value
ACI thrombolysis time (h)	4.0 ± 1.2	4.0 ± 1.2	<0.001
NIHSS score	12.0 ± 1.2	12.0 ± 1.2	<0.001
Systolic blood pressure before thrombolysis (mmHg)	156.0 ± 12.3	156.0 ± 12.3	0.568
Systolic blood pressure after thrombolysis (mmHg)	146.0 ± 12.3	146.0 ± 12.3	<0.001
Diastolic blood pressure (mmHg) before thrombolysis	86.4 ± 6.5	86.4 ± 6.5	0.742
Diastolic blood pressure after thrombolysis (mmHg)	81.4 ± 8.4	81.4 ± 8.4	0.921
Blood glucose concentration before thrombolysis (mmol/L)	8.4 ± 2.1	8.4 ± 2.1	<0.001
Blood glucose concentration after thrombolysis (mmol/L)	7.4 ± 0.8	7.4 ± 0.8	0.711

**Table 5:** Multivariate analysis of cerebral hemorrhage after ACI intravenous thrombolysis.

Factor	OR	CI	*P* value
ACI thrombolysis time	2.34	1.64–3.21	<0.001
NIHSS score	2.23	1.46–2.96	<0.001
Systolic blood pressure after thrombolysis	1.89	1.34–2.28	<0.001
Blood glucose concentration before thrombolysis	1.82	1.15–2.20	<0.001

## Data Availability

No data were used to support this study.

## References

[1] Liang Y., Song Q., Jiao Y. (2018). Cerebral microbleeds and the safety of anticoagulation in ischemic stroke patients: a systematic review and meta-analysis. *Clinical Neuropharmacology*.

[2] Alaa A., El D., Thouant P. (2019). Cerebral microbleeds and acute coronary syndrome: screening and progression under dual antiplatelet therapy. Proof of concept study - ScienceDirect. *Archives of Cardiovascular Diseases Supplements*.

[3] Zhai M., Wang J., Yu L., Fu X., Li L. (2017). Neutrophil and lymphocyte ratios for the predictive analysis of the prognosis in patients with acute cerebral infarction. *Chinese Journal of Cerebrovascular Diseases*.

[4] Pan L., Jin J., Huang R., Wang W., Chen Q. (2020). Application of transcranial Doppler in prognosis assessment of nerve function in patients with acute cerebral infarction after intracranial mechanical thrombectomy. *Zhonghua Wei Zhong Bing Ji Jiu Yi Xue*.

[5] Dong X. L., Xu S. J., Zhang L. (2017). Serum resistin levels may contribute to an increased risk of acute cerebral infarction. *Molecular Neurobiology*.

RETRACTED

[6] Papadopoulos A., Palaiopanos K., Protogerou A. P., Paraskevas G. P., Tsivgoulis G., Georgakis M. K. (2020). Left ventricular hypertrophy and cerebral small vessel disease: a systematic review and meta-analysis. *Journal of Stroke*.

[7] Yubi T., Hata J., Ohara T. (2018). Prevalence of and risk factors for cerebral microbleeds in a general Japanese elderly community. *Neurology: Clinical Practice*.

[8] Xia Y., Wang Y., Yang L. (2021). Incident cerebral microbleeds and hypertension defined by the 2017 ACC/AHA Guidelines. *Annals of Translational Medicine*.

[9] Meng T. T., Tian Z. Y., Xie X. L., Li T. T., Liu W., Gao Y. (2021). Systematic review and Meta-analysis of clinical efficacy and safety of Ginkgo Leaf Tablets in treatment of acute cerebral infarction. *Zhongguo Zhong yao za zhi = Zhongguo zhongyao zazhi = China journal of Chinese materia medica*.

[10] Zhou D., Xie L., Wang Y. (2020). Clinical efficacy of tonic traditional Chinese medicine injection on acute cerebral infarction: a bayesian network meta-analysis. *Evidence-based Complementary and Alternative Medicine*.

[11] Wu Z., Chen F., Yu F., Wang Y., Guo Z. (2018). A meta-analysis of obstructive sleep apnea in patients with cerebrovascular disease. *Sleep and Breathing*.

[12] Wang J., Fang K., Pang W., Sun J. (2017). Wind power interval prediction based on improved PSO and BP neural network. *Journal of Electrical Engineering and Technology*.

[13] Li D., Wu G., Zhao J., Niu W., Liu Q. (2017). Wireless channel identification algorithm based on feature extraction and BP neural network. *Journal of Information Processing Systems*.

[14] Zhang D., Huang D., Chong Z. (2017). Application of BP neural network based on genetic algorithm in the inversion of density interface. *Journal of Jilin University (Engineering and Technology Edition)*.

[15] Pan Q., Dong H., Han Q., Wang Y., Ding R. (2017). A computing method for attribute importance based on BP neural network. *Journal of University of Science and Technology of China*.

[16] Jin L., Chen M., Paediatrics D., Hospital L. (2017). Comparion between peripheral intravenous thrombolysis and deep vein catheter method applying in the treatment of acute deep venous thrombosis in lower limbs. *Medical Journal of Wuhan University*.

[17] Tambini D. T. R., Roberto (1999). Acyclovir for treatment of infectious mononucleosis: a meta-analysis. *Scandinavian Journal of Infectious Diseases*.

[18] Feick D., Valuenzuela C., Ahumada H. (2022). Re: effectiveness of non-benzodiazepine hypnotics in treatment of adult insomnia: meta-analysis of data submitted to the Food and Drug Administration. *BMJ*.

[19] Zhang X., Fang Q., Chen K. (2020). Distal perfusion cannulae in preventing limb ischemia in venous-arterial extracorporeal membrane oxygenation: a Meta-analysis. *Zhonghua Wei Zhong Bing Ji Jiu Yi Xue*.

RETRACTED

[20] Yu H., Gao L., Liao W., Zhang B., Pizurica A., Philips W. (2017). Multiscale superpixel-level subspace-based support vector machines for hyperspectral image classification. *IEEE Geoscience and Remote Sensing Letters*.

